# Endophytic Fungi and Secondary Metabolites of Rehmannia Glutinosa Based on Traditional Chinese Medicine Fingerprints

This article has been retracted.

**DOI:** 10.1155/2022/7701198

**Published:** 2022-08-30

**Authors:** Xiaotong Geng

**Affiliations:** School of Pharmaceutical Engineering, Xinyang Agriculture and Forestry University, Xingyang 464000, Henan, China

## Abstract

Research on the active components of medicinal plants has always been the focus of research, and research on the active components of medicinal plant endophytic fungi and their secondary metabolites has also attracted widespread attention. Endophytic fungi of medicinal plants are widely distributed and are ubiquitous in various biological groups in nature. Rehmannia glutinosa contains a variety of active ingredients, which are regarded as the top grade of Chinese medicinal materials. It is of certain significance to study endophytic fungi and their metabolites of Rehmannia glutinosa. In this paper, endophytic fungi and their secondary metabolites of Rehmannia glutinosa were studied using fingerprint technology, which initially understands the diversity of endophytic fungi in Rehmannia glutinosa. In this paper, the roots and leaves of Rehmannia glutinosa were used as experimental materials. The fungi were cultured in the medium, the fungi were isolated and purified by the tissue block method, the fungal growth of Rehmannia glutinosa in different parts was determined, and the types of endophytic fungi were identified by microscopic identification and fingerprinting. The isolated strains were tested for biological activity using oryza oryzae spores, and highly active strains were screened. Fermentation products of endophytic fungi were separated and purified by chromatography, and the structure of the compounds was identified by nuclear magnetic resonance spectroscopy. Through the above studies, the population structure of endophytic fungi of Rehmannia glutinosa was determined, 3 highly active strains were found, and the structures of 7 endophytic fungi metabolites were identified, of which 3 were newly discovered compounds.

## 1. Introduction

Endophytic fungi thrive inside healthy plants for part or all of their lives, but do not cause apparent syndromes of infection in the host vegetation. In recent years, endophytic fungi have been isolated from many medicinal plants, and the same or similar active ingredients as host plants have been isolated from these endophytic fungi. As a new source of many important medicinal ingredients, endophytic fungi can be industrially produced without the limitation of soil climate and resources, thus alleviating the shortage of medicinal sources. There are seldom research on endophytic fungi of Rehmannia glutinosa. Therefore, in this paper, the endophytic fungi and their secondary metabolites of Rehmannia glutinosa were studied using traditional Chinese medicine fingerprint technology.

Many scholars have studied endophytic fungi and their secondary metabolites in medicinal plants. El-Sayed et al. optimized the biological process of Astragalus endophyte and tested its anticancer activity [1]. Amorim et al. isolated antioxidant compounds from endophytic fungi of Luo Han Guo [2]. Kma et al. identified the active metabolites of Luo Han Guo endophytic fungi, and verified its anti-inflammatory and analgesic effects through experiments [3]. Zhu et al. extracted a new compound from the endophytic fungus of Safflower, and verified its bioprotective activity [4]. Abdou et al. studied the anticancer activity of the endophytic fungus Aspergillus sinigera in figs [5]. Although there are many studies on endophytes and their secondary metabolites, there are only a few studies on the endophytes of Rehmannia glutinosa.

Traditional Chinese medicine fingerprints can obtain chemical structures of traditional Chinese medicine compounds through certain analytical methods. It is a comprehensive and quantifiable identification method, which is widely used in the structure identification of traditional Chinese medicine compounds. Zhou et al. used spectroscopic and chromatographic methods to separate and identify the polysaccharide compounds in Rhizoma, Rhizoma [6]. The soft coral-derived fungus Penicillium has a variety of active metabolites, and Boulis et al. identified its chemical structure by fingerprinting, and found that the active metabolite has high antibacterial, anti-yeast, and cytotoxic activities [7]. Abd-Ellatif et al. carried out the structural identification of biologically active compounds of marine Streptomyces by spectrometry and chromatography, and tested their biological activities [8]. Ma et al. optimized the extraction process of diterpenoids from Euphorbia. The resulting extract under optimal extraction conditions identified 51 peaks, 2 of which were identified as novel compounds [9]. Yang et al. identified the structure of arabinogalacturonic acid in the peel of Chazhi orange by nuclear magnetic resonance spectroscopy [10]. Although traditional Chinese medicine fingerprints are widely used, the current research on traditional Chinese medicine fingerprints in the identification of compounds in Rehmannia glutinosa is not perfect.

In this paper, the endophytic fungi and their secondary metabolites of Rehmannia glutinosa were studied using traditional Chinese medicine fingerprint technology. In this paper, endophytic fungi were first cultured and isolated from tissue blocks to determine the growth characteristics of endophytic fungi. Then, the endophytic fungi species were identified by microscopic identification and fingerprinting. The isolated strains were then screened for active strains using the spores of M. oryzae, the active strains were cultured, and the compound structure of the fermentation product was identified by the fingerprint method, i.e., the secondary metabolites of endophytic fungi.

## 2. Experimental Materials, Instruments, and Reagents

### 2.1. Experimental Materials

The Rehmannia glutinosa used in the experiment came from the Rehmannia glutinosa planting base in Wenxian County, Henan Province. Healthy plants were selected and stored in a fresh-keeping bag at 4°C.

### 2.2. Experimental Equipment

The experimental equipment include DHP-9082 incubator (Shanghai Yiheng); YQX-LS-75SII autoclave (Shanghai Boxun); Motic2000 microscope (Motic); QYC-200 full temperature air shaker (Shanghai Fuma); SW-CJ-ID type ultra-clean bench (Suzhou purification); BSZ-100 type automatic collector (Shanghai Luxi); RE-52C rotary steamer (Shanghai Luxi); HHS-11-2 water bath (Shanghai Yukang); SHB-IIIA vacuum pump (Shanghai Yukang); Agilent1200 high performance liquid chromatograph (Agilent); ZF-20C UV analyzer (Shanghai Gucun); MP-250B mold incubator (Shanghai Nanrong); Multiskan MK3 enzyme label analyzer (Labsystems Dragon); KQ5200 B ultrasonic instrument (Kunshan).

### 2.3. Experimental Reagents

Yeast extract, glucose, sucrose, maltose, peptone, beef extract, agar, NaCl, *Na*_2_*SO*_4_, (*NH*_4_)_2_*SO*_4_, KCl, *KNO*_3_, *K*_2_*HPO*_4_, *MgSO*_4_, 7*H*_2_*O*, *CaNO*_3_, 4*H*_2_*O*, *MnSO*_4_, *H*_2_*O*, *F*_*e*_*SO*_4_, 7*H*_2_*O*, *NaNO*_3_, and *HgCl*_2_ were all of analytical grade (Sinopharm Group).

Silica gel (Qingdao Marine), chromatography column, methanol, dichloromethane, ethyl acetate (Shanghai Heqi), tritiated chloroform (Beijing Tengdayuan), tritiated methanol, pyridine, and dimethyl sulfoxide (Shandong Yantai) were also used.

## 3. Endophytic Fungi of Rehmannia Glutinosa

### 3.1. Isolation and Purification of Endophytic Fungi

1. Disinfection of plant tissue surfaces.
2. The Rehmannia glutinosa plants were classified according to blocks and leaves, rinsed off of dirt, dust, and other impurities on the surface with running water, respectively, and then the surface of the plants was disinfected. The steps are as follows: first soak the Rehmannia glutinosa plant with soapy water, and then rinse it with tap water until it is clean and has no foam. The rinsing process is about 1∼2 h. The roots and leaves are washed, cut into small pieces, and the plants are thoroughly disinfected with chemical solvents. First rinse with 75% alcohol for 3 minutes, then with sterile water 4 to 5 times, then with 0.1% mercury solution for 3 minutes, then with sterile water 5 to 6 times, and finally dry the surface with filter paper.
3. After surface disinfection of the plant tissues, 5 tissues were randomly selected and placed in Potato dextrose medium (PDM) medium for 10 minutes and then incubated at 28°C for 1–2 weeks to determine whether fungal growth occurs. If no colonies appear, bacteria have been removed; otherwise, there is the possibility of isolating surface bacteria; this experimental group should be discarded [11, 12].
4. Isolation and purification of endophytic fungi.
5. Experiment with the tissue block method, and the specific processing steps are as follows [13]:

Leaf: An appropriate amount of sterilized leaves were cut into small pieces of 2 cm × 2 cm, and inoculated into four mediums, respectively. Three leaves were placed in each plate, 20 plates of each medium, for a total of 80 plates.

Root tuber: Cut the sterilized root tuber into small pieces of about 1 cm × 1 cm × 1 cm, and inoculate them in four kinds of separation medium plates, respectively. Three roots were placed in each plate, 20 plates of each medium, for a total of 80 plates.

The inoculated medium was placed in a mold incubator. The state of the tissue block was observed every day. If new hyphae appeared on the tissue block, the hyphae were immediately picked and put into a new medium, and the colonies were gradually purified.

### 3.2. Microscopic Identification of Endophytic Fungi

After the purification of endophytic fungi, a small amount of spores were inoculated into PDM plates with an inoculating needle. Cultured at 28°C for 3 d, 7 d, and 10 d, the colony morphology was regularly observed, and the texture was examined under a microscope [14].

### 3.3. Fingerprints Assist in the Identification of Strains

The spores are planted in a PDM flat plate to obtain a culture solution, the culture solution is filtered to obtain mycelia, then put into an oven for drying, and the dried mycelium is pulverized. The culture solution was rotary-evaporated to the state of extract to obtain the crude extract; mycelia were extracted by the ultrasonic method with 20 ml methanol; all extracts were concentrated to 1 ml, filtered by a microporous membrane, and then detected by high-performance liquid phase chromatography. A Zorbax SB C-18 reverse column (150 × 3.0 mm, 3 *μ*m) was used with a Phenomenex C-18 pre-column (10 × 4.6 mm, 5 mm). The column oven was set to 30°C, acetonitrile was used for gradient elution, and 0.1% phosphoric acid aqueous solution was used as the mobile phase [15].

## 4. Secondary Metabolites of Endophytic Fungi of Rehmannia Glutinosa

### 4.1. Strain Screening

The preparation of the extract solution was carried out with sterile water. In the experiment, the M. oryzae spore suspension was added to the row of wells, and then 50 *μ*L was dropped into the first row of wells, which was pipetted evenly. Then, 50 *μ*L from the first row of wells was aspirated and added to the second row of wells and so on until the last row of wells. The wells with the extract solution added were placed in an incubator, and the morphology of oryzae spores was observed with a microscope [16].

The states of oryzae spores are represented by “4,” “3,” “2,” “1,” and “0”. Among them, “4” indicates that the spores of M. oryzae did not germinate, and the extract showed a strong inhibitory effect; “3” indicates that the spores germinated, but the hyphal morphology changed significantly, and the extract showed a strong deformation effect. “2”means that the spores germinate, but the hyphal morphology changes greatly, and the extract shows a moderate deformation effect. “1” indicates that the mycelium can grow, but the growth is hindered, and the extract shows weak activity; “0”indicates that the mycelium grows normally and the extract is inactive [17].

### 4.2. Detection of Secondary Metabolites

#### 4.2.1. Organic Solvent Extraction

The 5% concentration liquid seed liquid was inoculated into a 4 L culture flask to obtain a fermentation broth. The fermentation broth concentrated under reduced pressure was extracted three times with an equal volume of ethyl acetate, and then the ethyl acetate phase was collected. The ethyl acetate phase was rotary-evaporated in a rotary evaporator to the state of extract [18].

#### 4.2.2. Silica Column Gradient Elution

A chloroform/methanol series gradient developing agent was prepared; the gradients are 100 : 1, 50 : 1, 30 : 1, 20 : 1, 10 : 1, and 8 : 1, respectively; the sample solution was spotted on a silica gel plate, and then developed in different proportions of the developing agent, and the Rf value of the sample in different developing agents was calculated. In the experiment, a developing solvent with an Rf value of about 0.2 was selected, and the elution of the sample solution was carried out in a silica gel column.

#### 4.2.3. Sephadex LH-20-Purified Compounds

The eluted sample solution was eluted again by a Sephadex column, and two mobile phases, methanol and methanol/chloroform (1 : 1), were selected. An automatic receiver was used to automatically collect the eluted liquid, and the obtained solution was detected by thin layer chromatography. Since the sample is not lost, the column can be loaded repeatedly and the mobile phase can be changed to achieve a good separation effect.

#### 4.2.4. Structure Identification

The eluted high-purity compounds were rotary-evaporated to dryness, the dried samples were dissolved with deuterated reagents, and then transferred to NMR tubes. After dissolution, the solubility can be checked using a non-deuterated reagent, preferably deuterated chloroform. If it cannot be dissolved, consider deuterated methanol or dimethyl sulfoxide (DMSO), but samples dissolved in DMSO should not be recovered. After the sample was loaded, nuclear magnetic detection was carried out, and the spectrum of the obtained compounds was decomposed, and the C and H signals were assigned one by one [19, 20].

## 5. Findings and Discussion

### 5.1. Separation Effect of Different Media on Endophytic Fungi from the Roots and Leaves of Rehmannia Glutinosa

In this experiment, four different selective media, potato dextrose medium (PDM), Gau's medium, sand medium, and Martin's medium, were used to isolate and purify endophytic fungi. The results are shown in Table 1 and Figure 1.

It can be seen from the data that a total of 213 endophytic fungi were isolated from the 4 isolation media. Among them, there are 128 plants in tuberous roots and 58 plants in leaves. A certain number of root and leaf endophytes of Rehmannia glutinosa could be isolated from the four separation media, but the numbers and types were not exactly the same. The overall separation effect of the selected four media on the root and leaf endophytic fungi of Rehmannia glutinosa was: Sabouraud's medium > PDA medium > Gao's medium > Martin's medium. Sabouraud's medium was more suitable for the growth of Rehmannia endophytes than the other three media and could maximize the separation rate. Moreover, the strains isolated from Sabouraud's medium are also most of the other three, which can better show the diversity of endophytic fungi.

### 5.2. Comparison of Endophytic Fungi in the Roots and Leaves of Rehmannia Glutinosa

The infection status, diversity, and similarity of endophytic fungi in different strains and different parts were compared using five indicators of isolation rate, colonization rate, isolation frequency, diversity index (H′), and similarity coefficient.

(1) $$\begin{array}{c} \text{Separation Rate}=\frac{N\left(\text{strains}\right)}{N\left(\text{tissue blocks}\right)}. \end{array}$$

The isolation rate refers to the ratio of the total number of endophytic fungal strains obtained to the total number of tested plant tissue blocks. This metric measures the abundance of endophytic fungi in a particular plant tissue sample and the frequency of multiple infestations in the plant tissue sample.

(2) $$\begin{array}{c} \text{Colonization Rate}=\frac{N\left(\text{Infected tissue mass}\right)}{N\left(\text{tissue blocks}\right)}. \end{array}$$

Colonization rate refers to the percentage of tissue blocks infected by endophytic fungi to the total number of tissue blocks. This index can reflect the degree of endophytic fungus infection of different plants or different tissues of the same plant.

(3) $$\begin{array}{c} \text{Relative Frequency}=\frac{N\left(\text{Specific endophytic fungus}\right)}{N\left(\text{Total endophytic fungi}\right)}. \end{array}$$

Isolation frequency refers to the percentage of total isolates of a given endophyte in a sample, which can reflect the abundance of a certain endophytic fungi in the plant.

The diversity index is calculated by the Shannon-Wiener index formula as:

(4) $$\begin{array}{c} H^{\prime }=-\overset{K}{\underset{i=1}{\sum }}P_{i}\times \;\ln\;P_{i}. \end{array}$$

*k* is the total number of endophytic fungi species in the host, and *P*_*i*_ is the percentage of a given endophytic fungal strain in the total number of strains.

The similarity coefficient is calculated according to the Jaccard formula:

(5) $$\begin{array}{c} J=\frac{j}{a+b-j}. \end{array}$$

*j* is the number of endophytic fungi species shared by the two parts; *a* and *b* are the respective endophytic fungi species numbers of the two parts. According to the Jaccard similarity coefficient principle, *J* in the range of 0 to 0.25 indicates high dissimilarity; *J* in the range of 0.25 to 0.5 indicates moderate dissimilarity; *J* in the range of 0.5 to 0.75 indicates moderate similarity; and *J* in the range of 0.75 to 1 indicates high similarity.

The results of the isolation rate, colonization rate, and diversity index of endophytic fungi in the roots and leaves of Rehmannia glutinosa are shown in Table 2 and Figure 2.

For the colonization rate, separation rate, and diversity index of endophytic fungi, the tuberous root of Rehmannia glutinosa was higher than that of the leaf.

The endophytic fungi were isolated and identified from the roots and leaves of Rehmannia glutinosa, and 168 endophytic fungi were obtained. Among them, 112 strains produced spores, which were identified by morphological observation and they belonged to 10 genera. The specific results are shown in Table 3.

There are only four genera in common in roots and leaves, among which Fusarium is the dominant endophytic fungus in tuber roots and Alternaria is the dominant endophytic fungus in leaves. The similarity coefficient of endophytic fungi in tuber roots and leaves calculated by the formula was 0.5. According to the similarity coefficient principle, there were moderate differences in endophytic fungal composition between tuber roots and leaves.

### 5.3. Strain Screening Results

Screening experiments were carried out on 15 strains, and the detection activity of M. oryzae was shown in Table 4.

Among the 15 fungal strains, the activity of the culture liquid extract of 3 fungi was more significant, namely D7, D10, and D14, among which D10 had the best activity. The three strains were identified as Chaetomium sp., Verticillium sp., and Xylaria sp., respectively.

### 5.4. Structure Identification of Endophytic Fungal Metabolites

The secondary metabolites were detected, a total of 10 compounds were obtained, and the structures of 7 compounds were analyzed, among which compound 5, compound 6, and compound 7 were new compounds. The compound structures are shown in Figures 3–9.

The signal from ^13^C NMR (100 MHz, DMSO-d6) combined with the DEPT spectrum was assigned to *δ*: 132, 130.5, 122.7, 158.6, 113.4, 135.2, 200.0, 71.8, 29.9, 21.0.

The signal associated with ^13^C NMR (100 MHz, CDCl_3_) and the DEPT spectrum is assigned to *δ*: 69.3, 50.7, 197.6, 154.6, 103.8, 124.5, 129.3, 149.7, 115.5, 21.0, 50.93.

The signal associated with ^13^C NMR (150 MHz, CDCl_3_) and the DEPT spectrum is assigned to *δ*: 150.83, 145.01, 122.56, 102.89, 107.10, 137.13, 111.20, 161.02, 186.92, 149.01, 156.02, 107.33, 108.49.

The signal associated with ^13^C NMR (150 MHz, CD_3_OD) and the DEPT spectrum is assigned to *δ*: 105.0, 202.7, 143.4, 119.2, 125.6, 160.2, 131.5, 126.9, 129.3, 19.1, 116.9, 22.5.

The signal associated with ^13^C NMR (100 MHz, CDCl_3_) and the DEPT spectrum is assigned to *δ*: 108.5, 136.4, 153.7, 105.1, 153.9, 125.1, 165.3, 52.2, 160.5, 105.8, 146, 110.0, 163.3, 100.5, 171.1, 52.4, 56.4, 22.1.

## 6. Conclusion

In this paper, the endophytic fungi and their secondary metabolites of Rehmannia glutinosa were studied using traditional Chinese medicine fingerprint technology. In this paper, endophytic fungi were cultured and isolated from different parts of Rehmannia glutinosa through tissue blocks. It was found that Sabouraud's medium was more suitable for the growth of endophytic fungi of Rehmannia glutinosa, and the number and types of endophytic fungi in the roots of Rehmannia glutinosa were more than those in leaves. Then, the endophytic fungi were identified by microscopic identification and fingerprinting, and a total of 168 endophytic fungi were obtained. Among them, 112 strains produced spores, which were identified by morphological observation and belonged to 10 genera. Then, the isolated endophytic fungi were screened for strains, and three highly active strains were screened out. The selected active strain D10 was fermented and cultured. The chemical structure of the fermentation product was identified by chromatography and nuclear magnetic detection. A total of 10 compounds were obtained, and 7 compounds were analyzed, of which 3 compounds were new compounds.

## Figures and Tables

**Figure 1:** Isolation of endophytic fungi from Rehmannia glutinosa in different media.

**Figure 2:** Data analysis of endophytic fungi in the root and leaf of Rehmannia glutinosa.

**Figure 3:** Compound 1. ^1^H NMR (400 MHz, CDCl_3_) gave 8 hydrogen signals, including 3 aromatic hydrogen signals [*δ*: 7.59 (1H, d, *J* = 8.3 Hz, H-2), 7.01 (1H, dd, *J* = 8.4, 2.6 Hz, H-3),7.37 (1H, d, *J* = 2.6 Hz, H-5)], 1 methine signal [*δ*: 4.96 (1H, dq, *J* = 7.2 Hz, H-8)], and 2 methyl signals [*δ*: 1.45 (3H, d, *J* = 7.1 Hz, H-9), 1.92 (3H, s, H-10)].

**Figure 4:** Compound 2. ^1^H NMR (400 MHz, CDCl_3_) gave 8 hydrogen signals, including 3 aromatic hydrogen signals [*δ*: 6.79 (1H, d, *J* = 8.4 Hz, H-3), 6.32 (1H, dd, *J* = 8.4, 2.1 Hz, H-4), 6.18 (1H, d, *J* = 2.1 Hz, H-6)], 1 methoxy signal [*δ*: 3.66 (3H, s, H-9)], and 1 methylene signal [*δ*: 2.61 (2H, q, *J* = 5.6 Hz, H-7)].

**Figure 5:** Compound 3. ^1^H NMR (400 MHz, CDCl_3_) gave 11 hydrogen signals, including 3 aromatic hydrogen signals [*δ*: 3.84 (1H, m *J* = 7.2 Hz, H-2), 6.78 (1H, d, *J* = 8.4 Hz, H-6), 7.04 (1H, d, *J* = 8.4 Hz, H-7)], 1 methylene signal [*δ*: 2.05 (2H, d, *J* = 5.0 Hz, H-3)], 1 methoxy signal [*δ*: 3.5 (3H, H–5OCH3)], and 1 methyl signal [*δ*: 1.23 (3H, d, H-2)].

**Figure 6:** Compound 4. ^1^H NMR (600 MHz, CDCl_3_) gives 10 hydrogen signals, including 5 aromatic hydrogen signals [*δ*: 7.29 (1H, d, *J* = 8.71 Hz, H-3), 7.03 (1H, d, *J* = 8.70 Hz, H-4), 7.29 (1H, d, *J* = 8.41 Hz, H-5), 7,58 (1H, t, *J* = 8.42 Hz, H-6), 7.29 (1H, d, *J* = 8.41 Hz, H-7)], 2 active hydrogen signals [*δ*: 7.29 (1H, s, OH), 11.76 (1H, s, OH)], and 1 methoxy signal [*δ*: 3.93(3H, s, H–2OCH_3_)].

**Figure 7:** Compound 5. ^1^H NMR (600 MHz, CD_3_OD) gives 10 hydrogen signals, including 2 aromatic hydrogen signals [*δ*: 7.07 (1H, d, *J* = 8.3 Hz, H-4), 7.03 (1H, d, *J* = 8.3 Hz, H-5)], 2 methine signals [*δ*: 7.17 (1H, dd, *J* = 15.9, 1.3 Hz, H-1'), 6.37 (1H, dd, *J* = 15.9, 6.7 Hz, H-2')], and 2 methyl signals [*δ*: 1.85 (3H, dd, *J* = 6.7, 1.4 Hz, H-3'), 1.53 (3H, s, H-2)].

**Figure 8:** Compound 6. ^1^H NMR (400 MHz, CDCl_3_) gives 12 hydrogen signals, including 7 methine signals: [*δ*: 6.68(1H, dd, *J* = 10.5, 2.3 Hz, H-9), 6.24(1H, dd, *J* = 10.3, 3.1 Hz, H-8), 5.29(1H, t, *J* = 2.2 Hz, H-4), 4.31(1H, s, H-6), 3.91 (1H, dd, *J* = 5.7, 2.5 Hz, H-10), 5.74 (1H, m, H-1'), 5.49 (1H, m, H-2')], 1 methylene signal [*δ*: 4.79 (2H, t, H-3)], and 1 methyl signal [*δ*: 1.62 (3H, dd, *J* = 6.5, 1.5 Hz, H-3')]. The signal associated with ^13^C NMR (100 MHz, CDCl_3_) and the DEPT spectrum is assigned to *δ*: 171.5, 157.2, 69.13, 61.58, 71.88, 196.88, 1125.95, 149.69, 40.75, 88.13, 132.71, 126.25, 17.88.

**Figure 9:** Compound 7. _1_H NMR (400 MHz, CDCl_3_) gives 15 hydrogen signals, including 3 aromatic hydrogen signals, [c6.95(1H, s, H-2), 5.82(1H, s, H-10), 6.35(1H, s, H-12)], 3 methoxy signals, [*δ*: 3.74(3H, s, H–8OCH_3_), 3.5(3H, s, H–16OCH_3_), 3.5(3H, s, H–17OCH_3_)], and 1 methyl signal [*δ*: 2.10(3H, s, H-18)].

**Table 1:** Isolation of endophytic fungi from Rehmannia glutinosa in different media.

Number of endophytic fungi (strain)		Root	Leaf blade	Strains belong to several
PDM medium	Number of fungi	32	10	9
	The separation rate (%)	0.54	0.26	—
Kosher medium	Number of fungi	29	13	6
	The separation rate (%)	0.46	0.2	—
Schaefer's medium	Number of fungi	50	29	7
	The separation rate (%)	0.82	0.48	—
Martin medium	Number of fungi	17	6	5
	The separation rate (%)	0.27	0.11	—

**Table 2:** Data analysis of endophytic fungi in the roots and leaves of Rehmannia glutinosa.

Organ	Separation rate	Colonization rate	Diversity index
Root	0.51	0.56	1.72
Leaf blade	0.22	0.28	0.85
Amount	0.73	0.84	2.57

**Table 3:** Identification results of endophytic fungi from Rehmannia glutinosa.

Genus	Endophyte count (strain)	
	Root	Leaf blade
Rhizoctonia	12	5
Corynebacterium	1	0
Fusarium	40	11
Alternaria	13	14
Cytosporium	1	0
Ascocystis	9	0
Ascocystis	1	0
Piriformis	1	0
Penicillium	15	8
Trichoderma	5	0
Asporaceae	14	18
Total	112	56

**Table 4:** Oryzae detection activity.

Strain	Test concentration(*μ*g/ml)						
	500	250	125	62.5	31.3	15.6	7.8
D1	2	1	2	0	0	0	0
D2	2	2	2	2	0	0	0
D3	0	0	0	2	0	0	0
D4	2	2	1	1	0	0	0
D5	3	2	2	1	1	0	0
D6	2	1	1	1	0	0	0
D7	4	4	4	3	2	1	0
D8	3	2	2	1	0	0	0
D9	3	3	3	2	1	0	0
D10	4	4	4	4	4	3	3
D11	2	2	2	1	0	0	0
D12	2	2	1	0	0	0	0
D13	3	2	0	0	0	0	0
D14	4	3	3	2	2	1	0
D15	4	4	2	2	0	0	0
Blank PDM	0	0	0	0	0	0	0

## Data Availability

The data that support the findings of this study are available from the author upon reasonable request.
